The article "Multiobjective Optimization Design of Green Building Energy Consumption Based on Inorganic Thermal Insulation Nanomaterials" was retracted in 2023. Reasons: signs of a paper mill; suspected computer-generated content; unreliable results or conclusions; concerns about the data.

# Multiobjective Optimization Design of Green Building Energy Consumption Based on Inorganic Thermal Insulation Nanomaterials

**DOI:** 10.1155/2022/6993034

**Published:** 2022-06-24

**Authors:** Yuan Yuan, Songtao Li

**Affiliations:** Railway Engineering College, Zhengzhou Railway Vocational and Technical College, Zhengzhou, Henan 450052, China

## Abstract

In order to solve the problem that building engineering construction needs to consume a lot of energy and cause environmental pollution, which will pose a great pressure on urban resources and environment, this paper proposes that, in building engineering construction, appropriate green construction technology must be selected in combination with the actual situation, so as to effectively reduce the energy consumption of building engineering and improve the use efficiency of building engineering. Firstly, good thermal insulation nanomaterials are selected, which are cost-effective, safe, and nontoxic and has small thermal conductivity, large heat storage coefficient, stable chemical performance, and good construction performance. Secondly, it also needs to be selected according to the actual service life of the building. Because the current evaluation system is mostly aimed at the planning and design stage, and the structure occupies a large part in the building, for example, the impact on the construction period accounts for more than 50% and the impact on the cost accounts for 35%. Therefore, Duan Xiaorong and others established the grey cluster evaluation model of green building structure design based on the triangular whitening weight function. Finally, according to the relevant national regulations, this paper optimizes the design of green buildings based on the basic principles of energy conservation and emission reduction, high quality, and high efficiency.

## 1. Introduction

The construction industry, industry, and transportation industry have always been the three “big energy consumers” in China. According to the 2016 China Energy Statistics Yearbook, the total construction energy consumption of the construction industry in 2015 was about 910 million tons of standard coal, accounting for 26% of the total terminal energy consumption in China. The massive consumption of energy products has brought a series of social problems. In recent years, various climate disasters caused by the greenhouse effect occur frequently, and environmental problems have been put on the agenda of all countries, which has become an important problem to be solved urgently. Green building can save resources (energy, land, water, and material), protect the environment, and reduce pollution. They can provide people with a healthy, applicable, and efficient space to use. They are architecture living in harmony with nature. It follows the basic principles of sustainable development such as protecting the earth's environment, saving resources, and ensuring the quality of living environment. In China's green building evaluation standards, green building must be able to save resources (energy, land, water, material), protect the environment, and reduce pollution. This kind of building must provide people with a healthy, applicable, and efficient space to use.

The article "Multiobjective Optimization Design of Green Building Energy Consumption Based on Inorganic Thermal Insulation Nanomaterials" was retracted in 2023. Reasons: signs of a paper mill; suspected computer-generated content; unreliable results or conclusions; concerns about the data.

Among them, the research related to economic evaluation mostly starts from the macro and constructs the overall evaluation model from different angles, and there is no relevant standard for the economic evaluation of green buildings. Due to the complexity of green building itself, it is very difficult to evaluate its overall economy. Therefore, this paper selects the energy-saving project of green building to study its impact on the local economy of green building and carries out energy-saving optimization on this basis, so as to achieve the highest cost performance of green building energy-saving project. As a new concept in the construction industry, the development of green building in China has been restricted due to its implementation cost and available benefits. In particular, the uncertainty of incremental cost and incremental benefit makes developers often hold a conservative attitude towards the development of green buildings. As energy-saving projects account for a large proportion in green buildings, the choice of energy-saving schemes will directly affect the incremental cost and incremental benefit. Whether the economy of green building energy-saving scheme can be effectively evaluated will be related to whether developers can make scientific decisions. Inorganic living wall thermal insulation nanomaterials belong to class a noncombustible thermal insulation nanomaterials. They are composed of natural high-quality high-temperature resistant mineral nanomaterials as the main raw materials and natural plant protein fibers to optimize the combination of various solidified nanomaterials and inorganic modified nanomaterials. Due to the principle of flexible gradual change of thermal insulation nanomaterials and mutual integration of materials, we can truly realize environmental protection and energy-saving wall thermal insulation and phase change energy-saving products with high performance, such as thermal insulation, fire and water resistance, crack and sound insulation, light weight, and anti-falling off. The excellent characteristics of this nanomaterial are as follows: good thermal insulation performance, low thermal conductivity, and good thermal inertia performance. At the same time, it has the advantages of simple construction, safety, fire prevention, good crack resistance, high toughness, high heat resistance, environmental protection, and comfort, as shown in Figure 1.

The article "Multiobjective Optimization Design of Green Building Energy Consumption Based on Inorganic Thermal Insulation Nanomaterials" was retracted in 2023. Reasons: signs of a paper mill; suspected computer-generated content; unreliable results or conclusions; concerns about the data.

## 2. Literature Review

With the proposal of the concept of sustainable development, building energy conservation began to transform to green buildings. Green building is a building that follows the concept of sustainable development in the whole life cycle, saves resources, protects the environment and reduces pollution to the greatest extent, provides people with a healthy, comfortable, and efficient living environment, and lives in harmony with the surrounding environment. At present, China's green building has entered a rapid development stage, especially in the past two years, showing a rapid growth trend. At the same time, domestic academic research on green building has sprung up. At present, the academic research on green building has a wide range, but it mainly focuses on the construction of green building evaluation index system, the selection of evaluation methods, and the whole life cycle economic evaluation.

In order to enable developers to accurately understand the cost-effectiveness of green building projects and make scientific decisions, most scholars at home and abroad have established economic benefit evaluation models based on the whole life cycle theory through different methods. Liu and Guo combined the fuzzy comprehensive evaluation method on the basis of analytic hierarchy process and then constructed the evaluation model [1]. Wang believed that investors will reduce their willingness to invest because the economic benefits are not significant, but the free choice of investors makes green buildings have real options. Therefore, a real option evaluation method is proposed [2]. Sun et al. analyzed the incremental cost-benefit from the perspective of consumers and built a contribution decision-making model [3]. Chen et al. constructed a scenario analysis model to analyze the evolution path of incremental cost under different scenarios [4]. Hong et al. classified the costs according to the order of cost occurrence from the perspective of time and constructed the benefit estimation model. The case analysis shows that, through effective cost control, the economic benefits of green buildings can be improved, and their initial costs can be recovered within a certain time [5]. Hong et al. established the cost estimation model of each star of green building through the linear regression method and verified the reliability of the model [5]. Verma et al. also designed and implemented the software algorithm based on the theoretical construction of the cost estimation model [6]. Song et al. pointed out the key points of cost control through the identification of incremental cost [7]. Focusing on carbon emission costs and low-carbon technologies, foreign scholars put forward the 0-1 mixed integer programming method and constructed the cost decision-making model of green building. Liu et al. applied AANS to cost prediction and verified the feasibility of the model through multiple regression analysis [8]. Do and Ohsaki put forward a mixed integer optimization model to maximize the score of construction projects in LEED evaluation under the constraints of budget and design [9].

The article "Multiobjective Optimization Design of Green Building Energy Consumption Based on Inorganic Thermal Insulation Nanomaterials" was retracted in 2023. Reasons: signs of a paper mill; suspected computer-generated content; unreliable results or conclusions; concerns about the data.

To sum up, the incremental costs of green buildings with different evaluation methods, different grades, different building types, and different regions are different, but they can be avoided through scientific and reasonable scheme optimization and even produce benefits in the whole life cycle [10]. Domestic studies tend to evaluate the economic benefits of green buildings, that is, whether the scheme is feasible or not, while foreign scholars focus on the optimization of the economic benefits of green buildings, that is, under the established goal, through the allocation and optimization of various resources, minimize the construction cost, and maximize the economic benefits, so as to achieve the best performance of the building structure.

## 3. Use of Inorganic Thermal Insulation Nanomaterials in Green Buildings

### 3.1. Understanding of Inorganic Thermal Insulation Nanomaterials

#### 3.1.1. Relevant Regulations on the Wall Heat Transfer Coefficient in China

At present, there are many types of environmental protection and energy-saving wall thermal insulation nanomaterials in the market. Purchasers are required to make a reasonable choice by comprehensively considering the energy of nanomaterials and building conditions. In addition, it needs to be selected according to the actual service life of the building and so on. At present, there are many harmful substances in the wall thermal insulation nanomaterials in the construction industry, and the performance of thermal insulation, crack resistance, and dry shrinkage resistance is poor. In order to solve this problem, the rubber powder polystyrene particle thermal insulation slurry with good thermal insulation performance has been developed: the advantages of simple construction process, high strength, light weight, good volume stability, low cost, high heat storage coefficient, and low thermal conductivity [11]. Through the research and application of environmental protection and energy-saving wall insulation nanomaterials, many scientific and technological patents and scientific research achievements have been obtained. The state has also promulgated many relevant standards and regulations to ensure the quality and reasonable constraints of the construction industry and actively introduced foreign advanced technology, which has greatly improved the level of China's construction industry [12]. At present, the main problems to be solved of wall thermal insulation nanomaterials are as follows: the safety performance cannot be guaranteed, the thermal insulation and thermal insulation performance cannot be considered, the surface is prone to cracks, the functionality of thermal insulation nano materials is poor, and so on.

The article "Multiobjective Optimization Design of Green Building Energy Consumption Based on Inorganic Thermal Insulation Nanomaterials" was retracted in 2023. Reasons: signs of a paper mill; suspected computer-generated content; unreliable results or conclusions; concerns about the data.

China is generally divided into five zones, as shown in Table 1. In different zones, the heat transfer coefficient and thermal performance of the wall are different. In cold areas, it is necessary to consider cold prevention measures in winter for thermal insulation. The heat insulation and cooling performance in summer needs to be considered in hot areas, so there are higher limit requirements for the heat transfer coefficient of wall nanomaterials in extreme climate areas [13].

#### 3.1.2. Inorganic Active Wall Thermal Insulation Nanomaterials

The main reasons for cracks in the wall include too much shrinkage of the weighing or filling wall itself, insufficient performance of nanomaterials, poor construction technology, unscientific treatment of thermal bridges or joints, and insufficient external thermal insulation structure design. Dispersible polymer powder is a kind of good dry fluidity, which is the same as the modification mechanism of polymer emulsion to cement mortar [14]. After mixing with the cement mortar, the cement and polymer form a network structure. The surfactant in the lotion disperses the cement particles to increase the flow. At the same time, the hydrophilic colloid of the lotion can enhance the water retention performance of the mortar and prolong the setting time [15].

### 3.2. Application Advantages of Green Building Construction Technology

#### 3.2.1. Construction Advantages

The traditional construction methods and technologies are relatively backward, and the management is not in place, which has caused a lot of pollution to the environment and cannot meet the national standards. Green construction technology is a new type of construction technology. Compared with the original construction technology, it has higher construction efficiency and less impact on the environment. The use of some modern construction technology and management concepts in the construction process can not only effectively improve the construction efficiency of construction engineering but also ensure the construction quality of construction engineering [16]. Compared with the traditional technology, the green construction technology of construction engineering emphasizes the efficient utilization of energy and strengthening the construction environmental protection in the practical application, so that the construction engineering can not only meet the construction requirements but also take the road of sustainable development. It is necessary to fully ensure that all links of the construction shall be carried out in strict accordance with the green construction and make full use of the resources available onsite to maximize the use of nanomaterials and energy as shown in Table 2.

The article "Multiobjective Optimization Design of Green Building Energy Consumption Based on Inorganic Thermal Insulation Nanomaterials" was retracted in 2023. Reasons: signs of a paper mill; suspected computer-generated content; unreliable results or conclusions; concerns about the data.

#### 3.2.2. Water Saving Technology

Water resources on earth are limited. Protecting water resources and water ecology and paying attention to sustainable development are the development goals of building a water-saving city [17]. As a construction project with a large water user, water conservation is particularly important. In the construction process, the water-saving indicators should be included in the daily assessment management, and the water supply and drainage system of the construction project should be optimized. During the construction of the construction project, the domestic water and production water need to be measured separately. During the process, the collected rainwater or reclaimed water can be used to flush the onsite equipment and be recycled.

#### 3.2.3. Material Saving Technology

Saving nanomaterials has always been an important means for construction enterprises to control costs [18]. During the construction process, optimize the construction scheme, reasonably arrange the procurement plan of nano materials, strictly control the consumption of nano materials, improve the utilization rate of waste materials, improve the turnover times of nanomaterials, and actively promote new nanomaterials and new processes. For example, during reinforcement processing, optimize the batching in advance, use high strength instead of low strength, mechanical connection instead of binding connection, make rational use of waste reinforcement, and improve the utilization rate of reinforcement. During concrete processing, new nanomaterials such as fly ash, slag, and additives are used to reduce the amount of cement [19].

#### 3.2.4. Land Saving Technology and Construction Land Protection

As a key content in the construction design stage, land-saving construction should not be underestimated. In this regard, in the construction of construction projects, we should optimize the design of construction roads and properly arrange the setting of temporary facilities, which requires the construction unit to focus on planning the construction details and do a good job in the construction of temporary facilities. For example, the construction unit should reasonably plan the actual floor area of temporary houses, fences, construction sidewalks, and hard floors around the construction in combination with the requirements of the number of onsite construction personnel, construction building material reserves, construction production scale, and construction progress. When planning the land area of various infrastructure, the plane layout should be set up reasonably and scientifically, so as to ensure the actual needs of construction engineering construction. At the same time, it can also reduce the actual land area of waste and make the utilization rate of the land area of temporary facilities more than 85%, so as to ensure the rational use of land, reduce energy consumption materials and effectively expand the practical space area of housing construction [20].

The article "Multiobjective Optimization Design of Green Building Energy Consumption Based on Inorganic Thermal Insulation Nanomaterials" was retracted in 2023. Reasons: signs of a paper mill; suspected computer-generated content; unreliable results or conclusions; concerns about the data.

### 3.3. Evaluation Model of Incremental Comprehensive Benefits of Energy-Saving Design Scheme

Compared with traditional buildings, although the energy-saving design of green buildings will generate incremental design costs in the planning and design stage before construction and maintenance costs after project handover, it will bring energy-saving economic benefits, environmental benefits, and social benefits in the operation stage. The resulting incremental cost and incremental benefit, which is larger or smaller, need to be evaluated by model tools.

The so-called incremental comprehensive benefit refers to the difference between the incremental cost and incremental benefit of the construction project. Among them, incremental cost refers to the additional investment of green buildings compared with reference buildings (or benchmark buildings, i.e., nongreen buildings that only need to meet mandatory standards), mainly due to the application of energy-saving technology. Incremental benefits refer to the direct or indirect benefits brought by the reduction of operating costs during the operation of green buildings compared with the reference buildings [21]. Incremental comprehensive benefit is the difference between incremental benefit and incremental cost, as follows:

(1) $$\begin{array}{c} {\left(x+\alpha \right)}^{n}=\sum_{k=0}^{n}\left(\begin{array}{c} n\\ k \end{array}\right)x^{k}\alpha^{n-\kappa }, \end{array}$$

where *n* is the incremental comprehensive benefit; *x* is incremental benefit, including economic, environmental, and social benefits; and *n* represents incremental cost, mainly initial incremental cost. The specific composition is shown in Figure 2.

The article "Multiobjective Optimization Design of Green Building Energy Consumption Based on Inorganic Thermal Insulation Nanomaterials" was retracted in 2023. Reasons: signs of a paper mill; suspected computer-generated content; unreliable results or conclusions; concerns about the data.

## 4. Experimental Process and Analysis

### 4.1. Application of Inorganic Energy-Saving and Thermal Insulation Nanomaterials in External Wall Thermal Insulation

#### 4.1.1. Energy-Saving Curtain Wall

In the actual implementation of green building energy conservation project, glass curtain wall is commonly used. Among many types of glass curtain wall, the utilization rate of insulating glass is very high. In the process of installing insulating glass, we need to master the following contents:

*(1) Before the installation of the glass plate*. it is necessary to strictly detect the relevant quality of the glass plate, and strictly inspect the curing, size, and skid resistance of the structural adhesive. After all items meet the standards, the glass plate can be installed by fixing the Bluetooth plate. Before installing the glass plate on the beam, it is necessary to ensure that the plate surface and plate joints are aligned. If the gap between them is to be filled, cushion blocks need to be added. In the process of actual work, you can first find a similar wood semihard nanomaterial as the module, fix the position of the board, then remove the original module, and finally fix it with screws. (2) In the process of sealing the curtain wall, the gap can only be filled on the basis of the above work. After filling, glue should be injected for sealing. At this time, porous polyethylene foam can be used as the nanomaterial for filling. This study also uses this kind of nanomaterial for lining. The weather resistant silicone sealant can be selected as the nanomaterial for sealing, which can achieve the effect of rain proof and leakage proof. (3) The cleaning of energy-saving curtain wall is also very important. In the process of cleaning, blades and clean containers should be used to clean the glue joints and pollutants on the surface. After these works are completed, the energy-saving curtain wall should be maintained, so as to prolong the service life of energy-saving curtain wall [22].

#### 4.1.2. Application of Energy-Saving Glass and Special Roof Nanomaterials

In the construction process of some large buildings and public buildings, the probability of using traditional thermal insulation is very small. This large and public building can replace the lighting effect achieved by lighting by using new glass with strong daylighting ability. At the same time, this new glass has a good decorative effect. In addition, in the process of installing the outer wall of the building, the sunlight can be converted into heat or electric energy to illuminate the house or improve the indoor temperature. The glass daylighting roof is an effective case of converting solar energy into heat [23]. In addition, some well-known buildings in China, such as the water cube, also use some special building nanomaterials to convert sunlight into heat energy through their own gas film structure as shown in Figure 3.

The article "Multiobjective Optimization Design of Green Building Energy Consumption Based on Inorganic Thermal Insulation Nanomaterials" was retracted in 2023. Reasons: signs of a paper mill; suspected computer-generated content; unreliable results or conclusions; concerns about the data.

#### 4.1.3. Effect of Antirelease Agent on Chloride Ion Permeability of Concrete

Chloride ion erosion will weaken the passive film of reinforcement in concrete, aggravate the corrosion of reinforcement in concrete, and lead to the early failure of concrete durability. The electric flux of concrete decreases with the increase of strength grade. This shows that the addition of antisegregation agent has a certain adverse effect on the chloride ion penetration resistance of concrete, but the chloride ion penetration resistance of concrete in each group is still at the same level, that is, the Q-III level (1000 C ≤ Qs < 2000 C). Under the same strength grade, the addition of antisegregation agent increases the electric flux of concrete. With the increase of concrete grade, the increase of electric flux of concrete is greater. The existing concrete antisegregation agent has strong flocculation effect, which will lead to fast settling speed of concrete, instant loss of flow properties of concrete, and unfavorable workability of concrete. Therefore, an antisegregation agent for concrete and a preparation method thereof are proposed. The test and analysis provide important data support and reference for the application and popularization of antisegregation agent in concrete. The main conclusions are as follows:

1. Under the test conditions, adding antisegregation agent can effectively improve the segregation degree of C30 and C50 concrete and has no obvious negative impact on the compressive strength of concrete.
2. The addition of antisegregation agent leads to the increase of the total cracking area per unit area of concrete and the decline of early cracking resistance. Under the same strength grade, the addition of antisegregation agent has no obvious effect on the carbonation resistance of concrete.
3. Under each cycle, the strength and corrosion resistance coefficient of concrete added with compressive segregation agent increase, and the sulfate resistance of concrete is improved.
4. When the antisegregation agent is added, the electric flux of concrete increases and the antichloride ion permeability of concrete is weakened as shown in Table 3.

### 4.2. Setting of Buildings and Their Parameters

In order to obtain the energy saving of each energy-saving scheme, this paper sets up a reference building as its comparison benchmark. Through test simulation, each energy-saving scheme is compared with the benchmark scheme of the reference building to obtain its energy-saving, so as to provide data for the genetic algorithm solution later. The parameters of the reference building set in this paper meet the minimum requirements for buildings in hot summer and cold winter areas in the design standard for energy efficiency of public buildings. Among them, the outer wall enclosure structure adopts the following structure: 24 brick wall + 20 mm polystyrene board internal insulation, and its heat transfer coefficient is 0.564 W/m^2^K. The external window adopts ordinary hollow glass (hollow 12 mm), and the heat transfer coefficient is 2.4 W/m^2^·K, which just meets the energy-saving standard. The roof is made of 46 mm polystyrene plastic + 200 mm reinforced concrete floor + 20 mm mud lime mortar plastering, and the heat transfer coefficient is 0.475 W/m^2^·K. The air-conditioning and heating system adopts the air-cooled refrigerator + direct fired lithium bromide system [24]. The specific parameters are shown in Table 4 and Figure 4.

The article "Multiobjective Optimization Design of Green Building Energy Consumption Based on Inorganic Thermal Insulation Nanomaterials" was retracted in 2023. Reasons: signs of a paper mill; suspected computer-generated content; unreliable results or conclusions; concerns about the data.

### 4.3. Research on Green Building Evaluation Model

In order to make the evaluation results of green buildings more objective and scientific, domestic scholars mostly use the way of building mathematical models to evaluate green buildings based on the index system. At present, the widely used mathematical models include the following categories:

1. Extension comprehensive evaluation method
2. Based on the comprehensive evaluation index of each research object, the extension level is determined by calculating the extension index. The evaluation model of green building is established by using the multilevel extension theory, and quantitative analysis is carried out on the basis of qualitative analysis, so as to evaluate green building more scientifically. However, the biggest difference between the two is that the weight of primary and secondary indicators used in Qian qinzhen's model is determined by establishing the model through the correlation function, while Yabo and others simply use the weight in the green label and have only primary indicators.
3. Fuzzy analytic hierarchy process
4. In order to reduce the error caused by subjective evaluation, many scholars have conducted in-depth quantitative research on the weight of indicators. For example, Lei Yong, Wu Bing, and Li Xinjuan established a fuzzy comprehensive evaluation model of green buildings based on the analytic hierarchy process and conducted empirical research. On the basis of establishing the fuzzy comprehensive evaluation model, Bao Xueying and others put forward the concept of “building green degree,” which was then applied to empirical research to prove its reliability.
5. Grey clustering evaluation method
6. Because the current evaluation system is mostly aimed at the planning and design stage, and the structure occupies a large part in the building, for example, the impact on the construction period accounts for more than 50% and the impact on the cost accounts for 35%, Duan Xiaorong and others established the grey clustering evaluation model of green building structure design based on the triangular whitening weight function. Therefore, many domestic scholars apply this theory to the construction of evaluation model, propose to apply grey clustering evaluation model to the design stage of green building, establish evaluation model for building design, and conduct empirical research to prove its scientificity and reliability.
7. BP neural network evaluation method.
8. Evaluate green buildings faster and better. Li Xiaojuan and others also use the AHP and fuzzy theory to evaluate the collected green buildings and demonstrate their feasibility with examples.

The article "Multiobjective Optimization Design of Green Building Energy Consumption Based on Inorganic Thermal Insulation Nanomaterials" was retracted in 2023. Reasons: signs of a paper mill; suspected computer-generated content; unreliable results or conclusions; concerns about the data.

The above four evaluation methods have their own advantages and disadvantages. Among them, although the extension comprehensive evaluation model ensures objectivity and flexibility, it does not consider the relationship between levels. In fact, the indicators of this level may not be comparable, so the index weight determined from this needs to be verified. The grey clustering evaluation model is based on the grey theory. It has a good processing function for the lack of data and information, but the same subjectivity is strong. BP neural network evaluation method is an intelligent evaluation method, which can evaluate green buildings quickly and efficiently, but the biggest disadvantage of this method is that it needs a lot of data and information. In addition, its training and learning process is more complex. The current research is mostly a combination of one or several models, which still has a certain subjectivity. Therefore, future research needs to be more objective and scientific on the basis of deepening the index system and systematically determine the index weight. In addition, economic indicators should be included in the evaluation model to make green buildings truly fit the sustainable concept of coordinated development of economy and environment. To sum up, based on previous studies, this paper first discusses the factors affecting the development of green buildings and concludes that economic factors such as incremental cost and return on investment are the key factors hindering their development. Then, by summarizing and reviewing the relevant research on the incentive mechanism of green buildings, it is found that economic incentive has attracted much attention and is a quite effective incentive means, but how to grasp the incentive degree remains to be solved. Then, it summarizes and reviews the current research hotspot of green building at home and abroad, incremental cost-benefit research, which shows that there is a lack of research on scheme optimization in China.

The article "Multiobjective Optimization Design of Green Building Energy Consumption Based on Inorganic Thermal Insulation Nanomaterials" was retracted in 2023. Reasons: signs of a paper mill; suspected computer-generated content; unreliable results or conclusions; concerns about the data.

## 5. Conclusion

To sum up, with the rapid development of modern social economy, China's construction industry has developed greatly. Under the background of people's increasing living standards, the environmental protection requirements of construction projects are higher and higher, which urges the construction industry to strengthen the research on energy conservation and environmental protection. The thermal insulation work in building energy-saving engineering is directly related to the quality of building engineering. The application of inorganic thermal insulation nanomaterials in building energy-saving engineering has good application value.

## Figures and Tables

**Figure 1:** Energy consumption in green buildings.

**Figure 2:** Framework of incremental comprehensive benefits.

**Figure 3:** Relationship between gas film structure and thermal energy conversion.

**Figure 4:** Design scheme variables.

**Table 1:** Limits of building thermal zoning and wall heat transfer coefficient in China.

Thermal partition	Average temperature in the hottest month (°C)	Average temperature in the coldest month (°C)	Limit value of wall heat transfer coefficient, K (W/m^2^ K)	Remarks
Cold area A	＜−10	—	≤0.45	Heat protection is not considered in summer
Cold area B		—	≤0.50	
Cold area	0∼−10	—	≤0.60	
	>10	25∼30	≤1.0	
Hot summer and warm winter zone	>10	25∼29	≤1.5	Winter insulation is not considered
Temperate region	0∼13	18∼25		

**Table 2:** National building pollution standards.

Serial number	Target name	Target value
1	Construction waste	The construction waste produced per square meter shall not exceed 400 t
2	Noise pollution	Not more than 70 dB in the daytime and not more than 55 dB at night
3	Sewage discharge	The pH value is between 6 and 9, and the content of other pollutants is lower than the integrated wastewater discharge standard
4	Dust emission	The dust of structure construction shall not be greater than 0.5 m, and that of foundation construction shall not be greater than 1.5 m
5	Light pollution	No disturbance at night

**Table 3:** Effect of antisegregation agent on electric flux of concrete.

Project	A0	A1	B0	B1
Electric flux, Qs/C	1536.7	1569.9	1114.9	1221.5

**Table 4:** Parameter design of reference buildings.

Parameter name	Parameter engineering design value	Parameter specification limits
External wall heat transfer coefficient value	0.564	>3
	3.0	East 3.5; north and west 3.0
External window heat transfer coefficient	0.475	3.0
	0.5	West and south ≤5, east
Value of roof heat transfer coefficient	0.25	West and south ≤5
	2.1 3.0	≥4
Window wall ratio	1.0 ac/h	East, west, and south ≤5
Comprehensive shading coefficient scw	7 w/m	North and west 3.0
	1.07 c/h	West and south ≤5
Heating and air-conditioning system		West and south ≤5
Ventilation rate		
Lighting intensity		
Air tightness		

The article "Multiobjective Optimization Design of Green Building Energy Consumption Based on Inorganic Thermal Insulation Nanomaterials" was retracted in 2023. Reasons: signs of a paper mill; suspected computer-generated content; unreliable results or conclusions; concerns about the data.

## Data Availability

The data used to support the findings of this study are available from the corresponding author upon request.

## References

[1] Liu Z., Guo A. (2021). Application of green building materials and multi-objective energy-saving optimization design. *International Journal of Heat and Technology*.

[2] Wang X. (2021). Optimization design of green building landscape space environment based on VR virtual technology. *Journal of Physics: Conference Series*.

[3] Sun Z., Cao Y., Wang X., Yu J. (2021). Multi-objective optimization design for windows and shading configuration: considering energy consumption, thermal environment, visual performance and sound insulation effect. *International Journal of Energy and Environmental Engineering*.

[4] Chen B., Liu Q., Che H. (2021). Multiobjective optimization of building energy consumption based on BIM-DB and LSSVM-NSGA-II. *Journal of Cleaner Production*.

[5] Hong X., Shi F., Wang S., Yang X., Yang Y. (2021). Multi-objective optimization of thermochromic glazing based on daylight and energy performance evaluation. *Building Simulation*.

[6] Verma A., Prakash S., Kumar A. (2020). A comparative analysis of data-driven based optimization models for energy-efficient buildings. *IETE Journal of Research*.

[7] Song Y., Zhang H., Mo H. (2021). A LCA-based optimization method of green ecological building envelopes: a case study in China. *IOP Conference Series: Earth and Environmental Science*.

[8] Liu X., Zhang F., Sun Q., Zhong W. (2021). Multi-objective optimization strategy of integrated electric-heat system based on energy storage situation division. *IEEE Access*.

[9] Do B., Ohsaki M. (2021). Sequential sampling approach to energy‐based multi‐objective design optimization of steel frames with correlated random parameters. *Earthquake Engineering and Structural Dynamics*.

[10] Li Q., Wang Y., Zhang S., Xu W.-W., Bai L., Wang Z. (2020). Investigation and optimization of textured thrust bearings with spirally distributed dimples using multi-objective optimization method. *Industrial Lubrication and Tribology*.

[11] Yuvaraj N., Srihari K., Dhiman G. (2021). Nature-inspired-based approach for automated cyberbullying classification on multimedia social networking. *Mathematical Problems in Engineering*.

The article "Multiobjective Optimization Design of Green Building Energy Consumption Based on Inorganic Thermal Insulation Nanomaterials" was retracted in 2023. Reasons: signs of a paper mill; suspected computer-generated content; unreliable results or conclusions; concerns about the data.

[12] Jayakumar J., Nagaraj B., Chacko S., Ajay P. (2021). Conceptual implementation of artificial intelligent based e-mobility controller in smart city environment. *Wireless Communications and Mobile Computing*.

[13] Luo X., Liu Y., Liu X. (2021). Bi-level multi-objective optimization of design and subsidies for standalone hybrid renewable energy systems: a novel approach based on artificial neural network. *Journal of Building Engineering*.

[14] Talaei M., Mahdavinejad M., Azari R., Prieto A., Sangin H. (2021). Multi-objective optimization of building-integrated microalgae photobioreactors for energy and daylighting performance. *Journal of Building Engineering*.

[15] Monteiro S. A., Monteiro F. P., Tostes M. E., Carvalho C. (2020). Methodology for energy efficiency on lighting and air conditioning systems in buildings using a multi-objective optimization algorithm. *Energies*.

[16] Liu X., Ma C., Yang C., Diao Y. (2015). Power station flue gas desulfurization system based on automatic online monitoring platform. *Journal of Digital Information Management*.

[17] Mittelviefhaus M., Pareschi G., Allan J., Georges G., Boulouchos K. (2021). Optimal investment and scheduling of residential multi-energy systems including electric mobility: a cost-effective approach to climate change mitigation. *Applied Energy*.

[18] Salata F., Ciancio V., Dell’Olmo J., Golasi I., Palusci O., Coppi M. (2020). Effects of local conditions on the multi-variable and multi-objective energy optimization of residential buildings using genetic algorithms. *Applied Energy*.

[19] Huang R., Zhang S., Zhang W., Yang X. (2021). Progress of zinc oxide‐based nanocomposites in the textile industry. *IET Collaborative Intelligent Manufacturing*.

[20] Guo Z., Xiao Z. (2021). Research on online calibration of lidar and camera for intelligent connected vehicles based on depth-edge matching. *Nonlinear Engineering*.

[21] Javanmard M. E., Ghaderi S. F., Sangari M. S. (2020). Integrating energy and water optimization in buildings using multi-objective mixed-integer linear programming. *Sustainable Cities and Society*.

[22] Yuan Z., Zhou J., Qiao Y., Zhang Y., Liu D., Zhu H. (2020). BIM-VE-based optimization of green building envelope from the perspective of both energy saving and life cycle cost. *Sustainability*.

[23] Liu H., Zhang Z., Ma X., Lu W., Li D., Kojima S. (2021). Optimization analysis of the residential window-to-wall ratio based on numerical calculation of energy consumption in the hot-summer and cold-winter zone of China. *Sustainability*.

The article "Multiobjective Optimization Design of Green Building Energy Consumption Based on Inorganic Thermal Insulation Nanomaterials" was retracted in 2023. Reasons: signs of a paper mill; suspected computer-generated content; unreliable results or conclusions; concerns about the data.

[24] Zhang J., Ji L. (2021). Optimization of daylighting, ventilation, and cooling load performance of apartment in tropical ocean area based on parametric design. *Advances in Civil Engineering*.

